This article has been retracted.

# Long non-coding RNA HAL suppresses the migration and invasion of serous ovarian cancer by inhibiting EMT signaling pathway

**DOI:** 10.1042/BSR20194496

**Published:** 2020-03-04

**Authors:** Ke Wu, Lei Li, Lin Li, Dong Wang

**Affiliations:** 1 Gynecologic Cancer Center, Chongqing University Cancer Hospital and Chongqing Cancer Institute and Chongqing Cancer Hospital, Chongqing, China; 2 Department Pathology, West China Second Hospital, Sichuan University, Chengdu, Sichuan Province, China

**Keywords:** EMT, LncRNA HAL, migration, proliferation, serous ovarian cancer

## Abstract

**Objective:** To investigate the specific function of long non-coding RNA HAL in serous ovarian cancer (SOC) and to further clarify the regulation of HAL on EMT pathway.

**Materials and methods:** The expression of HAL and TWIST1 was detected by qRT-PCR. CCK8 assay, wound healing assay, transwell assay and flow cytometry were used to detect the HAL function on proliferation, migration, invasion and apoptosis in SOC cells. Western blot was used to calculate protein level of Vimentin, N-cadherin and E-cadherin. The effect of HAL on tumorigenesis of SOC was confirmed by xenograft nude mice model.

**Results:** HAL was significantly decreased in SOC tissues and cells. Overexpression of HAL inhibited the proliferation, migration and invasion of SKOV3 cells, but promoted apoptosis. Furthermore, overexpression of HAL decreased the mRNA and protein levels of TWIST1 via a binding between HAL and TWIST1. Forced expression of TWIST1 reversed the inhibitory role of HAL on SOC cells’ migration and invasion. The *in vivo* tumor growth assay showed that HAL suppressed SOC tumorigenesis with inhibiting EMT pathway.

**Conclusions:** Our research emphasized HAL acting as a tumor-inhibiting gene by regulating EMT signaling pathway, thus providing some novel experimental basis for clinical treatment of SOC.

## Introduction

Ovarian cancer, especially serous ovarian cancer (SOC), is one of the most common malignant diseases of the female reproductive system, with an overall 5-year survival rate of less than 35% [1,2]. Because of the location of SOC in pelvic cavity, the symptoms of SOC are hidden, many women have entered a progressive stage when the SOC was discovered [3]. The standard initial treatment for SOC is tumor cell reduction followed by platinum or paclitaxel chemotherapy [4]. Despite such aggressive treatment, recurrence and metastasis rates remain high [5]. Although other diagnosis and treatment methods have improved the treatment effect of patients, the long-term survival rate is still worrying. Traditional treatments have limited effectiveness because of lack understanding of the molecular mechanisms of disease progression [6]. Therefore, the priority is to explore the underlying mechanisms and develop effective treatment for SOC.

Long non-coding RNA is a kind of functional RNA molecule whose transcript length exceeds 200 nt, which can regulate gene expression at the epigenetic, transcriptional and post-transcriptional levels and widely participate in the physiological and pathological processes of the body [7,8]. In addition, a lot of data indicate that lncRNAs play an important role in the occurrence and development of cancer [9]. Studies have shown that lncRNA MALAT1 can be used as a biomarker, which is beneficial for the early diagnosis and treatment of the lung cancer [10,11]. LncRNAs also play an important role in the development of serous ovarian cancer. LncRNA H19 can promote the metastasis and invasion of ovarian cancer cells by inhibiting let-7 [12]. Silencing HOTAIR reduced the ability of epithelial ovarian cell carcinoma to metastasize and inhibited metastasis of ovarian cancer, which was possibly modulated by the EMT signaling pathway through MMP3 and MMP9 [13]. Recently, lncRNA HAL was reported to inhibit the breast cancer proliferation [14], which showed that silencing lncRNA HAL in MCF7 cells increased cell proliferation and impaired cancer stem cell proportion and function, resulting in decreased tumor grafting *in vivo*. However, the key role of lncRNA HAL in the development of serous ovarian cancer remains unknown.

Epithelial–mesenchymal transition (EMT) refers to the epithelial cells transforming into mesenchymal cells, thereby gaining the process of interstitial cell phenotype [15]. EMT was reported to be involved in embryonic development, tissue remodeling, wound healing, tumor metastasis and other pathological physiological process [16]. Meanwhile, EMT inhibited apoptosis and regulated the expression of transcription factors, such as Snail, Slug, ZEB1/2 and TWIST1/2 [17]. Studies have shown that cytokines in the microenvironment of ovarian cancer, including ET-1, TGF-β and EGF, can mediate the occurrence of EMT and activate regulate relevant signaling pathways to promote the progression of ovarian tumor [18–20]. However, whether HAL interacts with EMT pathway in serous ovarian cancer remains elusive. The purpose in our study was to clarify the specific function of lncRNA HAL in serous ovarian cancer and to further clarify regulation of HAL on EMT pathway.

## Methods and materials

### Clinical samples

Fresh cancer tissue samples and adjacent normal tissue samples were taken from 30 SOC patients undergoing surgical procedures at Chongqing University Cancer Hospital. All patients or their guardians provided written consent, and the Ethics Committee of Chongqing University Cancer Hospital.

### Cell culture and treatment

The cell lines were purchased from the Science Cell Laboratory. Cells were cultured in RPMI 1640 (GIBCO, U.S.A.) supplemented with 10% fetal bovine serum (Cromwell, U.S.A.) and 100 μl/ml penicillin and streptomycin (Sigma-Aldrich, U.S.A.) and placed at 37°C with 5% CO_2_. About 2 μg HAL plasmid or TWIST1 plasmid or its NC was transfected into SKOV3 cells with LipofectamineTM 2000 (Invitrogen, Carlsbad, CA, U.S.A.), respectively.

### RNA isolation and qRT-PCR

Total RNA was isolated from tissues or cells using Fast Pure Cell/Tissue Total RNA Isolation Kit (Vazyme, China). The concentration of RNA was examined by Nano-Drop 8000 Spectrophotometer (Thermo Scientific U.S.A.). Reverse transcription of RNA into cDNA used HiScript III RT SuperMix for qPCR (Vazyme, China). The relative expression levels of mRNAs were quantified by qRT-PCR with SYBR Green 1 (Vazyme, China). After circle reaction, the threshold cycle (*C*_t_) was determined and relative mRNA levels were calculated based on the *C*_t_ values and normalized to GAPDH level in each sample, and gene expression was calculated using 2^−ΔΔCt^ method.

### Protein isolation and Western blot

Total protein was collected from cells with RIPA lysis Mix. Western blotting assay was performed as previously described. Briefly, 60 μg protein extractions were loaded via SDS-PAGE and transferred onto nitrocellulose membranes (absin, China), then incubated with primary antibodies for 2 h at room temperature, then plated at 4°C overnight, the membranes were incubated in 5% non-fat milk blocking buffer for horizontal mode 3 h. After incubation with secondary antibodies, the membranes were scanned using an Odyssey, and data were analyzed with Odyssey software (LI-COR, U.S.A.). All primary antibodies were purchased from proteintech, including Bcl2 (12789-1-AP), bax (50599-2-Ig), caspase3 (19677-1-AP), vimentin (10366-1-AP), N-cadherin (22018-1-AP), E-cadherin (20874-1-AP) and GAPDH (60004-1-Ig).

### CCK8 assay

The proliferation was analyzed by Cell Counting Kit (Vazyme, China). A total of 5 × 10^5^ cells were seeded in 96-well cell plates, and added CCK-8 solution (Vazyme, China) at 0, 24, 48 and 72 h. And the cells were cultured for another 2 h, the OD value was measured at 450 nm using a microplate reader (Bio-Tek, U.S.A.).

### Wound healing assay

A total of 5 × 10^5^ cells were planted in a 6-well plate, and when the cells grew to fuse, two vertical parallel lines were drawn with 10 μl suction head against the ruler. The floating cells were washed with PBS and cultured in serum-free medium for 24 h. Images were taken at 0 and 24 h of cell culture, respectively.

### Transwell assay

Cell invasion was analyzed by transwell plates (Corning, U.S.A.) with 8 μm-pore size membranes with Matrigel. Cells in logarithmic growth phase were adjusted to 2 × 10^5^ cells/well of medium (without serum) and plated into the upper chamber insert pre-coated with 1 μg/μl Matrigel. Lower chamber was added with 500 μl of medium (with 10% FBS), and then incubate the chamber at 37°C for 48 h. The membrane was stained with 0.2% Crystal Violet and followed washed with 95% ethanal. The membranes with invading cells were observed by inverted microscope.

### *In vivo* tumor growth assay

Nude mice were purchased from Guangdong provincial experimental animal center for medicine. SOC cells (5 × 10^6^) transfected with HAL plasmid or NC were subcutaneously injected in right lower limb of the nude mice. Tumor size was measured every 5 days. After 30 days of injection, mice were intraperitoneally injected with 3% pentobarbital sodium and were killed by excessive anesthesia with a dose of 90 ml/kg, and the tumors were removed for follow-up study. The present study was reviewed and approved by the Institutional animal care and use committee of Chongqing University Cancer Hospital. The animal testing was conducted in laboratory of Chongqing University Cancer Hospital.

### Cell apoptosis assay

Cell apoptosis was calculated by Annexin V apoptosis kit (Beyotime, China), and the operating procedure was according to the kit instructions. A total of 5 × 10^5^ cells/ml were centrifuged and resuspended in 200 μl Binding Buffer with 10 ml Annexin V-FITC and 10 μl PI solution at room temperature in darkness for 15 min after which 300 μl Binding Buffer was mixed into the resuspension. Cell apoptosis level was detected within 1 h.

### Statistical analysis

The data are presented as means ± SEM. Statistical analyses were assessed with Student’s test and one-way ANOVA using GraphPad Prism 5.0. A value *P* < 0.05 was considered as statistically significant.

## Results

### LncRNA HAL is decreased in SOC clinical samples and cells

The level of the gene is the precondition for its regulatory function, so we first detected the expression of lncRNA HAL. As shown in Figure 1A, we collected cancerous and para-cancer normal tissue from 30 SOC patients, qRT-PCR was performed to test HAL level. We found that HAL expression was down-regulated in cancer tissues than that in adjacent normal tissues (Figure 1A). Meanwhile, we detected the level of HAL in normal ovarian epithelium IOSE80 and SOC cells SKOV3, OVcar3 and A2780. The results showed that HAL were decreased in serious of SKOV3 (Figure 1B).

**Figure 1:** Expression of HAL in SOC tissue and cells (**A**) The expression of HAL in glioma tissues (*n* = 30) and adjacent normal tissues (*n* = 30) determined by qRT-PCR (**P < 0.01). (**B**) qRT-PCR assay analyzed the expression of HAL in normal ovarian epithelium IOSE80 and SOC cells SKOV3, OVcar3 and A2780 (*P < 0.05).

### LncRNA HAL suppresses proliferation and promotes apoptosis of SOC cells

To further explore the function of HAL in SOC, we constructed HAL plasmid to force expression of HAL (Figure 2A). CCK-8 assay showed that overexpression of HAL significantly inhibited growth rate at 48 and 72 h than cells transfected with NC (Figure 2B). The apoptotic cells were detected by flow cytometry, and we found that HAL significantly accelerated SOC cell apoptosis both early and late apoptosis processes (Figure 2C). In accordance with flow cytometry data, Western blot also showed HAL remarkably promoted the expression of pro-apoptotic proteins Bax and caspase 3, but inhibited anti-apoptotic protein Bcl2 (Figure 2D).

**Figure 2:** Forced expression of HAL inhibits proliferation, but promotes apoptosis in SOC cells (**A**) The expression of HAL in SKOV3 cells after FGD5-AS1 plasmid or its NC transfection was determined by qRT-PCR (**P < 0.01). (**B**) CKK-8 assay was used to examine the cell growth at 0, 24, 48 and 72 h (*P < 0.05). (**C**) The apoptosis of cells was calculated by flow cytometry in SKOV3 cells (**P < 0.01). (**D**) Western blot was performed to detected the expression of apoptosis related peotien Bcl 2, Bax and caspase 3 (*P < 0.05).

### HAL inhibits migration and invasion of SOC cells

Because migration and invasion are the key steps for cancer progression, we then tested the role of HAL on migration and invasion ability in both normal and SOC cells. The wound healing suggested that HAL decreased the wound healing area, which exhibited a lower migratory ability in HAL transfected cells (Figure 3A,B). Transwell assay was used to test invasion. The results showed that HAL significantly reduced the cell invasive ability in normal and SKOV3 cells (Figure 3C,D).

**Figure 3:** HAL suppresses migration and invasion in normal and SOC cells FGD5-AS1 plasmid or its NC was transfected into IOSE80 SKOV3 cells. (**A** and **B**) Wound healing assay was used to detect cell migration (*P < 0.05). (**C** and** D**) Transwell assay was performed to check cell invasive ability (*P < 0.05).

### lncRNA HAL interacts with interacted with TWIST1 and inhibit EMT

EMT pathway plays an essential role in various types of cancers development, and TWIST1 is a key molecular of EMT pathway. And we speculated that HAL regulated SOC progression through TWIST1 and EMT pathway. To test our hypothesis, we detected the expression of TWIST1 when up-regulation or down-regulation of HAL. As shown in Figure 4A,B, the HAL significantly inhibited the mRNA and protein level of TWIST1, while silencing of HAL promoted TWIST1 expression. To clarify the relationship between HAL and TWIST1, we performed biotin–avidin affinity isolation system. And the qRT-PCR analysis revealed a binding of HAL to TWIST1 (Figure 4C,D). In addition, overexpression of HAL inhibited Vimentin and N-cadherin expression and promoted E-cadherin expression (Figure 4E), which indicated HAL could suppress EMT pathway.

**Figure 4:** LncRNA HAL interacts with TWIST1 and inhibits EMT SKOV3 cells were transfected with HAL or si-HAL or its NC, and the relative mRNA and protein expression of TWIST1 was determined by qRT-PCR (**A**) and Western blot (**B**) (*P < 0.05). (**C**) SKOV3 cells were transfected with biotinylated TWIST1 and then harvested for biotin-based affinity-isolation assay. TWIST1 was pulled down by HAL probe, and the expression of TWIST1 was analyzed by qRT-PCR (**P < 0.01). (**D**) HAL was pulled down by TWIST1 as analyzed by qRT-PCR (**P < 0.01). (**E**) Western blot was performed to detect the EMT-related protein expression of Vimentin, N-cadherin and E-cadherin (*P < 0.05).

### HAL suppresses the migration and invasion of SOC by inhibiting TWIST1

In order to confirm the function of HAL regulating TWIST1 in SOC cells, we cotransfected HAL with TWIST1 into SKOV3 cells. The transfection efficiency of TWIST1 was tested by qRT-PCR (Figure 5A). Overexpression of TWIST1 removed the inhibitory role of HAL on cancer cell growth (Figure 5B). And TWIST1 decreased apoptotic cell numbers when treatment with HAL plasmid (Figure 5C,D). Moreover, we found that forced expression of HAL facilitated the migration and invasion of SOC, while transfection with TWIST1 suppressed migration and invasion (Figure 5E,F).

**Figure 5:** LncRNA HAL inhibits proliferation, migration and invasion by inhibiting TWIST1 TWIST1 plasmid or its NC was transfected into SKOV3 cells. (**A**) qRT-PCR was used to detect the transfection efficiency of TWIST1 (**P < 0.01). (**B**) CKK-8 assay was used to examine the cell growth at 0, 24, 48 and 72 h (*P < 0.05). (**C**) The apoptosis of cells was calculated by flow cytometry in SKOV3 cells (**P < 0.01 vs. NC, ^#^*P* < 0.05 vs HAL). (**D**) Western blot was performed to detected the expression of apoptosis related protein Bcl 2, Bax and caspase3 (*P < 0.05, ^#^*P* < 0.05 vs HAL). (**E**) Wound healing assay was used to detect cell migration (*P < 0.05, ^#^*P* < 0.05 vs HAL). (**F**) Transwell assay was performed to check cell invasive ability (*P < 0.05, ^#^*P* < 0.05 vs HAL).

### HAL inhibits *in vivo* tumor growth in the nude mice

To determine the effect of HAL on tumorigenesis of SOC, we set up xenograft nude mice model. SKOV3 cells transfected with HAL or NC plasmid were subcutaneously injected into nude mice, and we measured tumor volume. The mice with HAL plasmid cells showed a smaller tumor volume, and tumors grew slower when forcing expression of HAL (Figure 6A). The tumors were isolated at 30 days after injection, HAL significantly decreased tumor’s weight than that in NC mice (Figure 6B). In addition, we isolated these tumor tissues and found that the expression of HAL was increased in HAL overexpression mice (Figure 6C). Moreover, HAL decreased the mRNA and protein level of Vimentin, N-cadherin and TWIST1, but increased E-cadherin expression in tumor tissues (Figure 6D,E).

**Figure 6:** LncRNA HAL inhibits *in vivo* tumor growth in the nude mice The nude mice were subcutaneously injected with SKVO3 cells (5 × 10^6^) transfected with HAL plasmid or NC in to the right flanks of the nude mice. (**A**) The tumor volume was assessed in the nude mice every 5 days (*P < 0.05). (**B**) Tumor weight was determined in the isolated tumors from the nude mice (*P < 0.05). (**C**) The relative expression of HAL was determined by qRT-PCR in the isolated tumor tissues (**P < 0.01). (**D**) qRT-PCR was performed to detect the relative mRNA expression of Vimentin, N-cadherin, TWIST1 and E-cadherin (*P < 0.05). (**E**) Western blot was performed to detect the relative protein expression of Vimentin, N-cadherin, TWIST1 and E-cadherin (*P < 0.05)

## Discussion

Serous ovarian cancer is a common malignant tumor in women, with a high incidence of gynecological malignancies and a low incidence of 5 percent of all malignant tumors [21]. Early detection and new treatment methods are important factors to reduce the occurrence and development of ovarian cancer, and the focus of clinical research [22]. At present, clinical treatment of serous ovarian cancer is mainly composed of surgical therapy and chemical therapy [23]. But due to the extensive basin celiac metastasis, the limitations of surgery and drug resistance and relapse after chemotherapy, the ovarian cancer patients with late 5-year survival rate is still stuck at 20–25% [24]. Therefore, seeking a new therapy for treatment of ovarian cancer is one of current hot research topics.

Recently, it have been shown that lncRNAs are widely involved in various biological processes regulation, including cell cycle, cell differentiation and many other life activities [25,26]. It is found that lncRNA has a great influence on the occurrence and development of liver cancer, laryngeal cancer, lung cancer and gastric cancer. LncRNA GMAN could interact with eIF4B and inhibited cancer cell apoptosis, thus promoted the survival and invasion of hepatocellular carcinoma [27]. In addition, LINC00460 acted as a sponge of miR-485 regulating Raf1, which facilitated proliferation, migration, invasion and EMT in papillary thyroid cancer [28].

In our study, we explored the expression of lncRNA HAL in SOC to clarify its function. Surprisingly, HAL was significantly decreased in clinical SOC tissues, and we also found a remarkable reduction of HAL in SOC cells. These data suggested that HAL might be involved in the development of glioma. To further investigate the role of HAL in SOC, we constructed HAL plasmid to force HAL expression. In accordance with expectation, HAL promoted apoptosis and inhibited the proliferation, migration and invasion of SKOV3 cells.

At present, the difficulty of multiple tumor treatments is the resistance of relapse and chemotherapy. Studies have pointed out that EMT signaling pathway is an important mechanism for the development of ovarian tumor [5,29]. Studies have shown that the BMP4-mediated signaling pathway led to morphological changes in tumor cells and enhanced cell adhesion, migration, and invasion by inducing EMT [30]. The EGFR signaling pathway inhibits the expression of miR-125a through the transcription factor PEA3, thereby promoting EMT and leading the poor prognosis [31].

And in this study, we surprisedly found that HAL inhibited the expression of EMT key molecular TWIST1. And biotin-avidin affinity isolation system showed there was a binding between HAL and TWIST1. Meanwhile, overexpression of HAL inhibited Vimentin and N-cadherin expression and promoted E-cadherin expression, which indicated HAL could suppress EMT pathway. Moreover, overexpression of TWIST1 removed the inhibitory effect of HAL on SOC cell proliferation, migration and invasion. The *in vivo* tumorigenesis of SOC got the same results, HAL exerted its tumor suppressive function via interacting with TWIST1 and inhibiting EMT pathway in SOC.

## Conclusions

In conclusion, our results showed that lncRNA HAL acted as a novel factor in regulation of SOC cell proliferation, invasion and metastasis via TWIST1 and controlling EMT signal pathway. In addition, there should be more clinical experimental basis for the clinical detection effect of HAL on SOC. On this basis, more prospective studies should be carried out to promote the early detection and treatment and prediction of the prognosis of SOC, which will benefit patients with SOC.

## Abbreviations

BMP4: bone morphogenetic protein 4
EGF: epidermal growth factor
EGFR: epidermal growth factor receptor
EMT: epithelial–mesenchymal transition
ET-1: endothelin-1
HAL: lncRNA-HAL
SOC: serous ovarian cancer
TGF-β: transforming growth factor-β
